The article "The National Children's Study Archive Model: A 3-Tier Framework for Dissemination of Data and Specimens for General Use and Secondary Analysis" was published in 2021. Journal: Front Public Health.

# The National Children's Study Archive Model: A 3-Tier Framework for Dissemination of Data and Specimens for General Use and Secondary Analysis

**DOI:** 10.3389/fpubh.2021.526286

**Published:** 2021-03-05

**Authors:** Peter K. Gilbertson, Susan Forrester, Linda Andrews, Kathleen McCann, Lydia Rogers, Christina Park, Jack Moye

**Affiliations:** ^1^Social & Scientific Systems Inc., Silver Spring, MD, United States; ^2^National Institutes of Health, Office of the Director, Bethesda, MD, United States; ^3^Eunice Kennedy Shriver National Institute of Child Health and Human Development, National Institutes of Health, Bethesda, MD, United States

**Keywords:** biological specimen bank, child health, data archive, data exploration, data sharing, environmental sample bank, information dissemination, longitudinal studies

## Abstract

The National Children's Study (NCS) Archive was created as a repository of samples, data, and information from the NCS Vanguard Study—a longitudinal pregnancy and birth cohort evaluating approaches to study influence of environmental exposures on child health and development—to provide qualified researchers with access to NCS materials for use in secondary research. The National Children's Study Archive (NCSA) model is a 3-tiered access model designed to make the wealth of information and materials gathered during the NCS Vanguard Study available at a user appropriate level. The NCSA model was developed as a 3-tier framework, for users of varying access levels, providing intuitive data exploration and visualization tools, an end-to-end data and sample request management system, and a restricted portal for participant-level data access with a team of experts available to assist users. This platform provides a model to accelerate transformation of information and materials from existing studies into new scientific discoveries.

**Trial Registration:** ClinicalTrials.gov Identifier: NCT00852904 (first posted February 27, 2009).

## Introduction and Background

The National Children's Study (NCS) Vanguard Study was a pilot for a nationally representative cohort of 100,000 U.S. children to be followed beginning before birth to adulthood (along with their parents) in a national longitudinal study of environmental (including physical, chemical, biological, and psychosocial) influences on child health and development, to be conducted by the *Eunice Kennedy Shriver* National Institute of Child Health Human Development (NICHD) in collaboration with the U.S. Centers for Disease Control and Prevention and the U.S. Environmental Protection Agency (1).

The Vanguard Study tested different recruitment strategies between 2009 and 2014. The Initial Vanguard Study (IVS) opened to accrual in 2009 in seven locations across the U.S. The IVS focused on recruitment through household enumeration, and used comprehensive data and sample collection procedures that were designed for the Main NCS (2). In November 2010, the IVS was succeeded by the Alternate Recruitment Substudy (ARS). The ARS was designed to evaluate three recruitment strategies: Direct Outreach, Enhanced Household Enumeration, and Provider-Based Recruitment (PBR). Each strategy was conducted in 10 study locations (3–5). Recruitment under the three ARS strategies ended in February 2012. The ARS was followed in June 2012 by another substudy, the Provider-Based Sampling (PBS) Substudy, which was conducted in three study locations (6). Overall, the PBS strategy proved most effective and cost efficient (7). In December of 2014, the Vanguard Study was discontinued by the National Institutes of Health (NIH) Director following the recommendations of a National Children's Study Working Group (8, 9).

To recruit Vanguard Study participants, over 74,000 women were screened to determine eligibility (Figure 1). At the close of the NCS Vanguard Study, more than 5,400 birth families had been enrolled and followed (Figure 1) in 43 counties within 31 states across the country (Figure 2). Over the course of the study, 5,608 children and their primary caregivers participated in at least one protocol-specified study visit, from pre-conception through pregnancy and birth up to 42 months of age (Figure 1).

**Figure 1:** NCS recruitment, enrollment, and study status flow by participant and activity.

**Figure 2:** NCS participating counties by recruitment strategy across the United States.

Data on a wide variety of health-related topics was collected by interview, self-administered questionnaires, and data collector generated case report forms. In total, 161 data collection forms, excluding form versioning (i.e., v1, v2, etc.), were utilized by the study for the IVS and ARS phases. These forms and the data they collected included pre-, peri-, and post-partum interviews, biological sample collection, environmental sample collection, physical examination, and neuropsychosocial and cognitive assessments. During active data collection, study centers submitted up to 700 datasets biweekly, totaling 4.1 terabytes of unique data by study end.

Nearly 19,000 unique biological and 4,000 unique environmental samples were collected from participants (women, fathers, and children) and their households across all study visit stages. From these a sample repository of more than 250,000 items was derived. Biological material collected includes blood, urine, saliva, breast milk, mucosal swabs, meconium, hair, nails, and placental tissue. Various air, dust, and water collections comprise the environmental samples. Serial sets of biospecimens were collected from women over several timepoints in pregnancy. Various combined sets of biological samples from mother/child dyads and some mother/child/father triads are represented.

The Vanguard Study, in addition to collecting data and samples, produced thousands of documents to support and facilitate study implementation. To effectively coordinate 40 locations across the country, each site worked from centrally created and maintained procedures and guidance documents. These documents were a combined effort of different teams of subject matter experts (SMEs) and defined the functions and implementation of the NCS. Each study task, such as data collection, had corresponding standard operating procedures (SOP), in-home study-visit and site workflows, training documentation, equipment maintenance guides, and adverse outcome documentation requirements. This documentation supporting the implementation of the NCS captured the many goals and challenges of executing any large, multicenter study.

With the Vanguard study's closure in 2014, the wealth of potential future research use represented by the existing data, samples, documentation, and knowledge of the NCS was recognized. The potential for data sharing was specifically noted in a 12/11/2014 NIH Director's statement indicating that “Data from the Vanguard Study should be archived and available upon request by investigators for secondary analyses” (10). Studies have shown that collaboration among researchers and the sharing of data not only promotes more robust research but also leads to faster translation of findings into clinical practice (11). The NIH therefore deemed that the NCS should continue as a scientific resource and sought to archive and make available the data and samples as quickly and completely as possible in accordance with the February 26, 2003 Final NIH Statement on Sharing Research Data (12).

The National Children's Study Archive (NCSA) core mission was to curate and maintain the information, data, and sample materials generated by the NCS Vanguard Study, and to make those products available for continued *de novo* analysis (9). The NCSA supported this mission from November 2015 to April 2020, after which the NCS data, following removal of HIPAA identifiers (13), is made available through the NICHD Data and Specimen Hub (DASH) (13) for continued research use beginning in early or mid-2020.

To support the NCSA mission, the NCS team developed the NCSA model to share the wide array of study protocols, procedures, instruments, and other products from the NCS, and to make available for scientific research the data and samples collected from women, fathers, and children for the NCS Vanguard Study. The objective of this report is to:

1. Describe the 3-tier NCSA model the NCS Archive developed to promote user access at a user appropriate level.
2. Describe the user-centric tools and resources developed for the NCSA model to facilitate the understanding of complex longitudinal study design and the resulting products.
3. Describe the evaluation framework the NCS archive used to support secondary analysis within the NCSA model.

## Materials and Methods

NCS leadership consulted experts within and outside the agency on various aspects of data archive design. The team reviewed existing data repository and data resource archives, including the Data and Specimen Hub (DASH, NIH/NICHD) (14), the Biospecimen Repository Access and Data Sharing program (BRAD, NIH/NICHD), the Prostate, Lung, Colorectal, and Ovarian Cancer Screening Trial (PLCO, NIH/NCI) and the Biologic Specimen and Data Repository Information Coordinating Center (BioLINCC, NIH/NHLBI) (15) to determine best archive and repository solutions for dissemination of NCS Vanguard Study data. The NCS reviewed data sharing practices and procedures of the National Health and Nutrition Examination Survey (NHANES; CDC/NCHS), National Database for Autism Research (NDAR; NIH/NIMH), and the NICHD Population Dynamics Branch. Some of the criteria evaluated included data specifications, data documentation and discovery tools, remote analysis functionality, and privacy protection measures.

Because of the complex and unique nature of the NCS Vanguard Study's design and conduct, and to meet the need for further data curation, the NCS Archive was created as a study-specific resource rather than a component of an existing data repository. As a separate resource, the NCS Archive could support carry-over research from the NCS Vanguard Study, release study data and information on a rolling basis, provide immediate support for secondary research projects, and share experience upon which other national cohort studies like the Environmental influences on Child Health Outcomes (ECHO) (16) and All of Us studies (17) could build.

While NCSA planning, development, and implementation predated establishment and publication of the FAIR (Findable, Accessible, Interoperable, Reuseable) Guiding Principles for scientific data management and stewardship (18), these principles were anticipated in the functional requirements that were established for the system.

Data security and privacy requirements were developed to ensure establishment of adequate controls to protect the privacy of the participants and ensure the security of the data as required by the Department of Health and Human Services (http://www.hhs.gov/ocio/policy/index.html#Security) and by the Federal Information Security Modernization Act of 2014 and Federal Information Security Management Act of 2002 (FISMA) (19).

System design requirements were established to achieve specific desirable characteristics, including:

- Flexible—quickly and efficiently accommodate evolving requirements
- Comprehensive—support an extensive range of data analysis functions
- Integrated—provide interoperability across data sources
- Reliable—assure function under all conditions
- Secure—employ stringent security controls to prevent inappropriate information disclosure and possible data loss, while ensuring that the right information is provided to the right people
- Private—ensure data privacy and integrity despite technological evolution
- Maximum access to data by researchers while maintaining FISMA standards
- User-focused and User-friendly—tailored to a variety of data users
- Reduction of long-term risks and lifecycle costs

Definition of functional requirements incorporated input, review, and comment from data users as part of the process. Key functional requirements of the NCSA are summarized below for various elements of the Archive.

Data curation, preparation, and documentation for easy reuse:

- Create analytic data files and all documentation including user guides, data dictionary, and code books, to be made available for the general research community and in accordance with Section 508 of the Rehabilitation Act of 1973 (20).
- Harmonize all analytic data files across multiple protocol versions to the extent possible in terms of file structures, variable naming, labeling, coding, and formatting.
- Produce final data files that meet Data Documentation Initiative (DDI) standards.
- Produce a comprehensive list of all biological and environmental samples in inventory with documentation of informed consent available for each NCS universal participant identifier.
- Readily update the inventory based on NCS sample repository use reports.
- The sample inventory and result data should be linkable to other analytic data at the participant level.

Restricted Use Data (RUD) file construction:

- Remove sensitive variables to comply with the NIH data privacy protection requirements
- Perform other data manipulation techniques to reduce disclosure risks
- Develop and implement specifications to minimize participant disclosure risk
- Produce data documentation needed by data users, including analytic limitations imposed by removal of personal identifiers.

Support tools development:

- Create new data discovery and cohort discovery tools based on existing applications such as the NCS Workbench and NCS Knowledgebase
- Provide links to questionnaires and data collection instruments and materials
- Develop and construct data item level crosswalks to facilitate data use
- Incorporate search capabilities into these data user tools
- Provide web-based analysis tools for end data users
- Produce data tables and charts that summarize participant characteristics or key findings from analytic files

Archive user support services:

- Support requests for data access (microdata, specimens)
- Produce other custom data files
- Development and maintenance of common linking identifiers to integrate NCS data with external sources while maintaining participant confidentiality
- Support linkages to laboratory data
- Disclosure review of researcher produced analysis outputs and tables
- Support for publication submission

Requirements for multiple levels of data access:

- Provide a limited set of carefully de-identified data files containing key variables which can be downloaded by users to be analyzed on their own equipment, as an inexpensive method to access key variables from the NCS.
- Provide a secure enclave wherein users can access more sensitive, partially de-identified data and conduct analyses within the enclave, with no ability to download any microdata (individual-level data).

## Results

The NCSA model shares information using a 3-tier approach built on the “principle of least privilege” and augmented with user driven content tools (Figure 3). Each tier is intended to allow users to identify the Study information and the available data at their level of need. Need-based access has three goals—first, to streamline the process of data absorption; second, to allow the user to drive meaningful discovery; and third, to allow targeted use of limited analytic and support resources. Key to the NCSA model is the leveraging of user self-service opportunities. Through either documentation or system tools information, information access is democratized. Users drive access and understanding of a study on their own, thereby reducing the resource requirements of Archive support staff and SMEs.

**Figure 3:** NCSA Model Access Tiers.

### Tier 1: Public Access

The Public Access tier is intended for the general population to allow persons interested in the research to learn about the content without unnecessary technical detail. For the NCS, public access meant access to the public portion of the NCS Archive website and a NICHD hosted web page. Users had access to a study description (21), a history of the study, descriptions of the data and samples available, and information about the ongoing archive activities. Users were provided a mechanism to gain registered access and a mechanism to contact the NCS Archive with questions or inquiries.

Public access for the NCS additionally meant highlighting a selection of scientific works for both informational and aspirational purposes. Publications based on NCS data presented in journals and at conferences were made available together with a series of data briefs, which are concise summaries of selected data from the NCS Archive, with comparisons to other widely recognized sources of similar data (Table 1).

**Table 1:** Published NCS data briefs.

**NCS data briefs**
Analysis of Alcohol and Tobacco Prevalence and Cessation before and during Pregnancy in the NCS
Breastfeeding and Autism Spectrum Disorder (ASD) in the National Children's study
Breastfeeding in U.S. Infants—How NCS and CDC National Immunization Survey Data Compare
Physical measures among children in the National Children's study
Risk factors affecting maternal health and pregnancy collected in the NCS vanguard study

This allowed sharing of previous work completed using NCS data and highlighted opportunities for new or continued research. As a federally funded program, it was important for NCS to make tangible results available to the general population. As a value-added component, the NCS Archive created and freely provided teaching databases comprised of child-level and health topic-related modules (22). The teaching databases were derived from real data collected during the NCS Vanguard Study. They were created for academic use only and not intended to be suitable for use for publication. The teaching databases offer a ready-made database system with examples for various statistical models, including repeated measures analyses, to supplement classroom instruction and for use in student projects.

### Tier 2: Registered Access

The registered access tier of the NCSA model provides the next level of data access privilege to users interested in a study. Registered access makes available resources to promote and cultivate new ideas for further exploration of existing data or samples, as well as providing detailed documentation of the study and the study's experiences. In exchange for the access to new information, a user must register and attest to responsible stewardship of the information provided.

For the NCS Archive, restricted access to the site required completion of a demographic registration form (Table 2), consent to adhere to the NCS Vanguard data user agreement (Table 3), and registering a login service account. Registered users gained access to all publicly available Study information and data files, the site's protocol and data self-service tools, and the proposal management system for requests to access restricted study data and other stored materials in Tier 3.

**Table 2:** Registration collected demographic elements and requirements.

**Demographic element**	**Required**
Name	Yes
Professional Title	
Institution	Yes
Department	
Email Address	Yes
Phone Number	Yes
Fax Number	
Physical Address	Yes
Website Address	

**Table 3:** NCS data use agreement terms.

	**Agreed terms**
1	To use NCS resources for the purposes of archiving and accessing data obtained from scientific research with the intent of data sharing and reuse, and to notify the NCS Administrator of any breach in use
2	To use NCS data for scientific research in an institution with an approved assurance from the Department of Health and Human Services Office for Human Research Protections, and to not use the data for commercial purposes (or sell the data obtained from NICHD)
3	To preserve and protect the confidentiality of, and not attempt to identify, any individuals or households in the data
4	That archived data are provided without warranty or liability of any kind
5	To notify the NCS Administrator of any errors discovered in the archived data
6	To establish safeguards to prevent unauthorized viewing or release of NCS information or data
7	To comply with any charges that may apply for various services offered by NCS
8	To ensure that the means of access to NCS (such as passwords) are kept secure and not disclosed to anyone else
9	That personal data submitted by you are accurate to the best of your knowledge and kept up to date by you
10	That personal data provided by you may be used for administrative management of NCS and for reporting purposes with the goal of improving services offered by NCS
11	That any breach of the User Agreement could lead to termination of your access to the services
12	[Privacy Act Notification] that information collected from the Recipient, as part of the data use agreement or data request forms, may be made public in part or in whole for tracking and reporting purposes. This Privacy Act Notification is provided pursuant to Public Law 93-579, Privacy Act of 1974, 5 U.S.C. Section 552a. Authority for the collection of the information requested below from the recipient comes from the authorities regarding the establishment of the National Institutes of Health, its general authority to conduct and fund research and to provide training assistance, and its general authority to maintain records in connection with these and its other functions (42 U.S.C. 203, 241, 289l-1 and 44 U.S.C. 3101), and Section 301 and 493 of the Public Health Service Act. These records will be maintained in accordance with the Privacy Act System of Record Notice 09-25-0200 (https://oma.od.nih.gov/forms/Privacy%20Documents/PAfiles/0200.htm) covering “Clinical, Basic and Population-based Research Studies of the National Institutes of Health (NIH), HHS/NIH/OD.” The primary uses of this information are to document, track, and monitor and evaluate the use of the NCS Archive, as well as to notify interested recipients of updates, corrections or other changes to the NCS data The Federal Privacy Act protects the confidentiality of some NIH records. The NIH and any users that are provided access to the NCS Archive will have access to the information collected by the NIH from the Recipient, as part of the data use agreement or data request forms for the purposes described above. In addition, the Act allows the release of some information without the Recipient's permission; for example, if it is requested by members of Congress or other authorized individuals. The information collection requested is voluntary, but necessary for obtaining access to data and samples in the NCS Archive
13	To complete NCS data user training

The NCS Archive developed several self-service tools to explore the study operational information and sample size data for participants, biospecimen, and environmental samples (Table 4), to facilitate meaningful evaluation and consumption of the large amount of available NCS data. These tools transfer the ability to identify and confirm potential research opportunities from the Archive support staff to the interested user, preemptively answering potential inquiries.

**Table 4:** NCS archive self-service tools and domains of coverage.

**Self-service tool**	**Domain**
Protocol browser	Operational
Instrument and dataset inventory	Operational
Variable locator	Operational, Sample size
Participant explorer	Sample size
Sample explorer	Sample size

One challenge to understanding the NCS Vanguard is a study design that involves multiple sequential study protocols—the 2009–2010 IVS Protocol and the 2011–2014 ARS Protocol. Each protocol included participant visits across multiple life stages (pre-conception, prenatal, perinatal, postnatal). The ***Protocol Browser*** tool was developed to allow users easily to assess the content and timing of study evaluations undertaken by NCS participants in either protocol. The tool is a visual representation of study events experienced by participants within each protocol, displayed by life stage, study visit, and data collection instruments administered (Figure 4). The tool can display one or both protocols simultaneously to allow comparisons.

**Figure 4:** NCS Protocol Browser.

With numerous Study visits for each protocol across multiple life stages, IVS with 14 visits and ARS with 16, the NCS ended up fielding 161 different instruments (IVS 97, ARS 64). To manage the dissemination of these instruments, the ***Instrument and Dataset*** ***Inventories*** tool (Figure 5) was developed to display a list of available instruments by protocol and subject domain. Instruments are made available in PDF format, unless copy restrictions apply, and interested users can view the in-line variables notation. Additionally, the number of variables and records in each corresponding dataset is identified.

**Figure 5:** NCS Archive Instrument Inventory.

From these instrument datasets and other constructed analytic files, the NCS Archive generated nearly 14,000 variables. To quickly evaluate what variables are available with how many data points or responses for a given area, the ***Variable Locator*** tool (Figure 6) was created. This tool provides for free text variable search of all data in the NCS Archive. A user who might enter the term “sleep” into the Variable Locator would be provided a list of all sleep-related variables and questions, together with frequency counts of respondents, valid responses, legitimate skip responses, and records in the dataset. The Variable Locator allows users to filter results further by using Boolean search terms (“AND,” “NOT,” and “OR”). Researchers can use the Variable Locator tool to identify readily what potential the NCS Archive data may hold for their intended research.

**Figure 6:** NCS Archive Variable Locator.

Once researchers have identified operational components of interest—datasets, instruments, or variables—knowing the potential sample size is crucial to evaluate the feasibility of their planned research. The ***Participant Explorer*** tool allows users to interrogate metadata-level NCS participant and study participation information. Users of the Participant Explorer tool can determine participant counts by various categories separately or in combination, such as type of participant (woman, child, father), data collection timepoint (prenatal, perinatal, postnatal), demographic variables (race, ethnicity, education level, marital status), etc. Data for fathers, for example, can be categorized by age, education, race/ethnicity, other demographics, and study activity (Figure 7). Each variable in the Participant Explorer allows a researcher to narrow the target population to reflect a researcher's specific needs and interest.

**Figure 7:** Participant Explorer for father participants in the IVS phase.

In similar fashion, the ***Sample Explorer*** allows users to develop sample size estimates based on the inventory of biological and environmental samples collected from women, children, and fathers who participated in the NCS (Table 5). The Archive initially held over 250,000 individual biospecimens and 4,600 individual environmental samples. This extensive sample collection made the Archive a significant resource of materials for laboratory research, while the Sample Explorer provided a method to explore those samples in context and detail. Like the Participant Explorer, the Sample Explorer allows researchers to determine the number and type of primary or derivative biological and environmental sample material available by various demographic categories, type of participant, study visit, etc. Researchers can use the Sample Explorer to determine counts of samples available from the specific type of participant (e.g., infants, pregnant women, etc.) of most interest to them. Once the available sample types, sample demographics, and sample size information are known, researchers can develop specific proposals to request those data and samples for their research.

**Table 5:** NCS Biospecimen and Environmental Samples available by Collection Period.

		**Collection period**		
**Sample category**	**Sample Type**	**Prenatal**	**Perinatal**	**Postnatal**
**Biological**	Blood	X	X	X
	Breast Milk		X	X
	Cord Blood		X	
	Hair	X		
	Meconium		X	
	Nail	X		
	Placenta		X	
	Saliva	X		X
	Umbilical Cord		X	
	Urine	X	X	X
	Vaginal Swab	X		
**Environmental**	Air—Fine particulate matter	X		X
	Dust—Plate	X		
	Dust—Vacuum	X		X
	Dust—Wipe	X		
	Infant formula		X	
	Water—Pesticides	X		
	Water—Pharmaceuticals	X		

Within the NCSA model, the user driven content framework and tools enable researchers to target specific populations, topic areas, and types of biological or environmental samples to determine quickly the feasibility of a research proposal. The research tools empower researchers to explore study information and to develop and refine their research ideas independent of SMEs. The tools help to decrease the knowledge gap between Archive staff and general users and allow Archive staff to provide expert knowledge and experience on narrowly targeted questions about potential research.

Once researchers determined the feasibility of using NCS resources, the Archive leveraged a user-driven electronic proposal submission system to submit, process, and review researcher requests for data alone or for combined data and biological and/or environmental samples to pursue their scientific objectives. Electronic forms collect information such as title, requesting investigator, institution, other users for whom approved access is requested, and a detailed plan of research (rationale, main hypothesis, and proposed research aims) (23). Additionally, the sample request form collects data about shipping accounts, laboratory contact information, specific sample information, and testing parameters such as target analytes and assay platforms.

Along with the completed request form, potential researchers can submit documentation of institutional review board (IRB) determination or review and approval, documentation of funding availability, and letters of institutional support. Other documents such as curriculum vitae (CV) or biosketch are encouraged but not required. When a research request is submitted, the researcher receives notification via email of receipt and processing. The NCSA model framework thus allows user-driven discovery, ideation, and data request submission.

Submitted requests next pass through a stringent multi-step review. Requests are first screened by Archive staff for completeness and clarity. Analysts then assess the practical feasibility of request fulfillment. Preliminary data frequencies are run and availability of suitable samples in sufficient quantities and amounts is reviewed, according to information submitted in the request form. In parallel, a review is conducted to assure compliance with regulatory and ethical requirements, evaluate appropriateness for the intended purpose of the specific data and any samples requested, and determine whether the research plan is consistent with the NCS informed consent. Discussions between the researcher, Archive staff, and NICHD staff may be needed to determine how best to fulfill a request. The potential impact on the repository inventory also is taken into consideration when samples potentially suitable for a request are identified, and an assessment is made whether the selected samples (including quantity, volume, concentration, etc.) and proposed assay methods are suitable for the planned research. If the requested data or samples are unavailable, or research plans are deemed unacceptable, immediate notification of investigators is provided, with further processing of the request suspended.

After the initial review, the request and the preliminary feasibility analysis enter a queue for formal review by an NCS Data Access Committee (DAC) composed of NICHD scientists and *ad-hoc* subject matter experts. Requests can be reviewed by individual DAC members immediately and are not dependent on a formal meeting. Members are given an initial 10-day review window and have access to review all submitted request materials within the electronic request system. Members use standard evaluation criteria for review (Table 6) and can share thoughts amongst themselves in a restricted discussion board.

**Table 6:** NCS archive request review criteria.

**Criterion**	**Description**
Scientific expertise	Should the request be reviewed by external experts? Reviewers are asked to identify external experts if appropriate
Scientific merit	Is the research plan well-designed and likely to provide meaningful results?
Significance	Does the request address an important problem? Will it improve scientific knowledge, technical capability, and/or clinical practice?
Approach	Is the overall strategy, methodology, and analytic plan well-reasoned and appropriate?
Statistical power	Is statistical power adequate to meet the stated aims?
Sample suitability	Are any samples requested suitable for the proposed research?
Sample use merit	Does the proposed research warrant the use of any requested biological or environmental samples?
Sample-data linkage	Is sample-associated data needed to achieve the stated goals available?
Investigator qualifications	Are the investigators qualified to perform the proposed research?
Environment	Are adequate institutional support, equipment and other physical resources available to the investigators?

If the DAC has questions, needs clarification, or needs additional information, the Archive staff work with the researcher to provide the requested information. Once the review is completed, the requester is notified of the review outcome by Archive staff. Accepted requests continue along the data access process, while unapproved research requests are returned to the requester with explanation.

The next step in the data access process is completion of a Research Materials Distribution Agreement (RMDA). The RMDA is a contract between the Principal Investigator of the proposed research, their institution, and the NICHD. It ensures that all parties are signatories and aware of the agreed terms for accessing participant-level NCS data, and it confirms their commitment to the policies and procedures put in place to protect the rights of NCS participants and institutions. Once the RMDA is executed, researchers move to the third tier of access.

### Tier 3: Restricted Access

The restricted access tier of the NCSA model is the most highly restricted level. It provides access and interaction with participant-level data collected during the NCS Vanguard Study and is the tier at which Archive staff interact with identifiable data. For the NCSA, investigators enter the restricted access tier through a secure virtual environment, known as the Researcher Portal.

For the Researcher Portal, Archive staff create a personalized virtual machine with statistical software that the researcher accesses through security authentication requirements (two-factor token, username, and password). Staff remain in communication with the researcher to ensure successful access to the Portal. The Portal allows for a spoke-hub distribution model whereby archive staff can centrally coordinate the flow of information between geographically disparate researchers.

Archive staff populate the researcher's folder with the requested data and coordinate all aspects of sample distribution, including sample selection based on proposal-defined characteristics. As an incentive to return laboratory test result data to the Archive and thereby expand available Archive data resources, participant-sample linkages are withheld until results are returned. With the NCSA model the limited technical support on tier 1 allows staff to provide concierge support on tier 3 for researchers. Staff work closely with the researcher to ensure that the Archive can provide for successful completion of a project. This includes assisting with any questions about how the data were processed, providing additional data analysis, transferring output, programs, and summary files in and out of the Portal, linking supplemental files such as geographic characteristics or other data to NCS data, and assisting with writing and reviewing articles for publication, including adherence to NCSA data publication guidelines (Table 7). Prior to release of information once the research project is complete, Archive staff performs a disclosure review of any information to be transferred out of the Researcher Portal to the researcher, to assure that the information meets disclosure standards.

**Table 7:** NCS archive data publication guidelines.

	**Data Publication Guidelines**
1	Access to personally identifiable information (PII) is not permitted
2	Absolutely no individual level data should be published or made publicly available
3	No attempts at re-identification shall be made
4	All presented count data is of *N* ≥ 10 (this refers to both data presented and data derivable from a presented table). If an *N* < 10 is presented or derivable, aggregation of cells or the presentation of percentages (without an *N*) are acceptable fixes
5	Derived counts refer to tables where multiple rows and columns are presented allowing a careful reader to infer a smaller count
6	Names of geographic areas smaller than the primary sampling unit are not mentioned
7	Any maps of geographic areas provided do not depict secondary sampling units (or smaller)
8	Employers, hospitals, providers, or industries are not named as residing in sampled areas
9	Potential or enrolled participant demographics or health status are not described at the individual level

From its opening in November of 2015 through December 2019, there were over 20,000 visits to the NCS Archive (Table 8) by users from more than 50 different countries. Those visitors spent on average 6 min and 27 s on the site browsing the available resources. This highlights the strength of the NCSA model, where the resources for user self-service are both available and utilized. Of those visits, 476 moved from Tier 1 access to Tier 2 by registering with the site. Using the exploratory tools and accessing study documents, those users submitted 59 research requests to gain access to NCS data and specimens, 44 of which started or completed research within the NCSA Tier 3 framework. These researchers represent 43 academic, non-profit, commercial, and government organizations/institutions. The researchers, 60 percent of whom have more than 10 years of scientific experience, range from undergraduate and graduate students to research scientists, professors and medical doctors. Over fifty peer reviewed publications have resulted from use of NCS Vanguard data and specimens (1–7, 24–69) as of January 2021.

**Table 8:** NCS archive site visit metrics.

	**Time period**					
	**11/2/2015–12/31/2015**	**1/1/2016–12/31/2016**	**1/1/2017–12/31/2017**	**1/1/2018–12/31/2018**	**1/1/2019–12/31/2019**	**Summary values**
Visits	458	4,290	4,586	6,900	4,369	20,873
Average visit duration (s)	332	412	436	392	313	387
Page views	2,167	21,414	27,367	34,772	17,337	103,057
Downloads	180	3,070	2,960	3,770	3,018	12,998

## Discussion

Data sharing is becoming an imperative for U.S. scientific research funding agencies. Recent calls for mandated data sharing (70) were followed by the October 29, 2020 announcement of the Final NIH Policy for Data Management and Sharing (71). The new policy establishes the requirements of submission of Data Management and Sharing Plans, applies to research funded or conducted by NIH that results in the generation of scientific data, and links compliance to funding actions. Related notices provide considerations for selecting a data repository, desirable characteristics for all data repositories, and additional considerations for repositories storing human data (72). NIH promotes the use of established data repositories because deposit in a quality data repository generally improves the FAIRness (Findable, Accessible, Interoperable, and Re-usable) of the data. The National Library of Medicine provides a useful listing of NIH Data Repositories at https://www.nlm.nih.gov/NIHbmic/nih_data_sharing_repositories.html.

The widely acknowledged benefits of data sharing must be balanced against the paramount need to protect privacy and maintain confidentiality of research participants (73). The human scientific research enterprise relies absolutely upon trust between research participants and researchers. Public trust in research is built over decades but can be destroyed in seconds and take lifetimes to repair, as exemplified by episodes such as the U.S. Public Health Service Syphilis Study at Tuskegee (74). Specific challenges for information security and privacy protection are presented by datasets like those of the NCS that incorporate chronological or geographic information that can be linked to other datasets with potential to reidentify individual research participants. Creative solutions to these challenges are illustrated by the secure data enclave models of the NCHS Research Data Centers (75), of which the Tier 3 restricted access level of the NCSA model represents a virtual equivalent.

The three-tier NCSA framework developed by the NCS Archive provides a model that allows researchers to evaluate information and data at a level appropriate for them, protects the rights of research subjects, and provides interactive support to researchers for specific research goals and outcomes.

The NCSA example represents a new model for adding value to large cohort studies after they close or even during their conduct and can serve as a model for effective and interactive data platform development, with tools and processes that empower users, protect research participants, and reduce the distance between data and knowledge.

## Peer Review

External peer review of the National Children's Study was carried out by the National Academy of Sciences in 2008^1^, in 2013^2^, and in 2014^3^.

## Data Availability Statement

The datasets and other materials supporting the conclusions of this article are available in the National Children's Study Archive (https://ncsarchive.s-3.net) through the spring of 2020. In 2020, the NCS Archive data files will be available in the NICHD Data and Specimen Hub (DASH) (https://dash.nichd.nih.gov/study/228954) after removal of HIPAA identifiers.

## Ethics Statement

Written informed consent was obtained from all participants and the study protocol was approved by the Institutional Review Boards (IRBs) of NICHD and each Vanguard Study institution. All procedures involving human subjects were approved by the Institutional Review Board of the Eunice Kennedy Shriver National Institute of Child Health and Human Development (Office for Human Research Protections Database IRB00000008 - National Insts Hlth - NICHD - IRB #8, FWA00005897).

## Author Contributions

PG and JM prepared the final manuscript. All authors participated in the design and conduct of the project, analysis and interpretation of the data, manuscript preparation and review, and read and approved the final manuscript.

## Conflict of Interest

PG, SF, LA, KM, and LR were employed by the company Social and Scientific Systems Inc. The remaining authors declare that the research was conducted in the absence of any commercial or financial relationships that could be construed as a potential conflict of interest.

## Footnotes

^1^National Research Council and Institute of Medicine. (2008). *The National Children's Study Research Plan: A Review*. Panel to Review the National Children's Study Research Plan. Committee on National Statistics, Division of Behavioral and Social Sciences and Education. Board on Children, Youth, and Families and Board on Population Health and Public Health Practice, Institute of Medicine. Washington, DC: The National Academies Press.

^2^National Research Council and Institute of Medicine. (2013). *Design of the National Children's Study: A Workshop Summary*. Nancy Kirkendall, Rapporteur. Committee on National Statistics, Division of Behavioral and Social Sciences and Education. Board on Children, Youth, and Families, Institute of Medicine. Washington, DC: The National Academies Press.

^3^National Research Council and Institute of Medicine. (2014). *The National Children's Study 2014: An Assessment*. Panel on the Design of the National Children's Study and Implications for the Generalizability of Results, G.J. Duncan, N.J. Kirkendall, and C.F. Citro (Eds). Committee on National Statistics, Division of Behavioral and Social Sciences and Education, and Board on Children, Youth, and Families, Institute of Medicine. Washington, DC: The National Academies Press.

## Abbreviations

ARS: Alternate Recruitment Substudy
BioLINCC: Biologic Specimen and Data Repository Information Coordinating Center
BRAD: Biospecimen Repository Access and Data Sharing program
CDC: Centers for Disease Control and Prevention
CV: Curriculum Vitae
DAC: Data Access Committee
DASH: Data and Specimen Hub
ECHO: Environmental influences on Child Health Outcomes
FISMA: Federal Information Security Management Act
HIPAA: Health Insurance Portability and Accountability Act
IRB: Institutional Review Board
IVS: Initial Vanguard Study
NCI: National Cancer Institute
NCHS: National Center for Health Statistics
NCS: National Children's Study
NCSA: National Children's Study Archive
NDAR: National Database for Autism Research
NHANES: National Health and Nutrition Examination Survey
NHLBI: National Heart, Lung, and Blood Institute
NICHD: National Institute of Child Health and Human Development
NIH: National Institutes of Health
NIMH: National Institute of Mental Health
PBR: Provider-Based Recruitment
PBS: Provider-Based Sampling
PDF: Portable Document Format
PLCO: Prostate, Lung, Colorectal, and Ovarian Cancer Screening Trial
RMDA: Research Materials Distribution Agreement
RUD: Restricted Use Data
SME: Subject Matter Expert
SOP: Standard Operating Procedures.
